# Apolipoprotein E polymorphisms are associated with ischemic stroke susceptibility in a Northwest China Han population

**DOI:** 10.1042/BSR20171088

**Published:** 2017-11-29

**Authors:** Li-li Zhao, Gang Su, Li-xia Chen, Qi Yan, Xue-ping Wang, Wei Yuan, Lei Wang, Zhen-chang Zhang

**Affiliations:** 1 Department of Neurology, The Second Hospital of Lanzhou University, Lanzhou, Gansu 730030, China; 2 School of Basic Medical Sciences, Lanzhou University, Lanzhou, Gansu 730030, China

**Keywords:** Apolipoprotein E, gene polymorphisms, Ischemic stroke, Neurology

## Abstract

Ischemic stroke (IS), the leading neurology cause of death and disability worldwide, is influenced by gene polymorphisms. To explore the association between IS and Apolipoprotein E (*APOE*) gene polymorphisms, a case–control study containing 513 IS patients and 514 controls without IS was conducted in a Northwest China Han population. MassARRAY iPLEX system was applied to determine the *APOE* polymorphisms according to the alleles of two single nucleotide polymorphisms (SNPs) of *APOE*, rs429358, and rs7412. The results showed that rs429358 and rs7412 were in Hardy–Weinberg equilibrium (HWE) in both cases and controls groups. *APOE* ε4 allele, ε4/ε4 genotype, and ε4-containing genotypes were associated with IS. According to the results of Trial of ORG 10172 in Acute Stroke Treatment (TOAST) classification system, *APOE* ε2 allele, ε4 allele, and ε4/ε4 genotype were associated with large artery atherosclerosis IS subtypes. In addition, the results also indicated that the ε4 allele related to undetermined IS and ε4/ε4 genotype was related to small vessel disease IS. Compared with subjects with non-ε4-containing genotypes, the total cholesterol (TC) and low-density lipoprotein (LDL) level in blood and the proportion of cardiopath history were higher in all subjects with ε4-containing genotypes. Besides, the triacylglycerides (TG) level in blood was higher in controls with ε4-containing genotypes. In conclusion, in a Northwest China Han population, *APOE* ε4 allele was associated with blood lipid level. The TC and LDL levels were the independent risk factors for IS. *APOE* was a risk gene for IS, but not independent, especially for large artery atherosclerosis IS.

## Introduction

Stroke is the leading neurology cause of death and disability worldwide [1]. In China, the annual mortality rate of stroke is approximately 157 per 100 000, which has accounted almost 20% of all death. China has 2.5 million new stroke cases and 7.5 million stroke survivors in each year [2]. According to the research conducted by China National Stroke Registry, ischemic stroke (IS) was a predominant stroke subtype in China, which accounted for 66.7% [3]. As a complex heterogeneous disease of multiple etiologies and major clinical manifestations, IS not only associated with kinds of traditional risk factors but also influenced by the gene polymorphisms [4]. Therefore, many candidate genes which may be related to IS, for example Apolipoprotein E (*APOE*), methylenetetrahydrofolate reductase (*MTHFR*), histone deacetylase 9 (*HDAC9*), human leukocyte antigen (*HLA*) and so on, have been studied by researchers [5–8].

*APOE* gene locates on 19q13.2 and encodes an important protein which has vital functions in lipid metabolism. The *APOE* gene has three alleles (ε2, ε3, and ε4) that encode three isoforms (E2, E3, and E4) protein. The three alleles of *APOE* gene form six genotypes (ε2/ε2, ε2/ε3, ε2/ε4, ε3/ε3, ε3/ε4, and ε4/ε4), of which, the ε3/ε3 is the most common genotype in China. The three isoforms of APOE protein have one amino acid difference at positions 112 and 158, and have variance of protein function and affinity to lipid and receptors [9]. Compared with ε3, ε4 allele was associated with increased risk for a variety of pathologies, for instance, neurological conditions, cerebrovascular diseases, Alzheimer’s disease [10], IS [11], and atherosclerosis [12]. ε2 allele was reported as a protective factor with a lower risk for dementia [13], and it was also associated with longevity [14,15]. However, studies on the association of *APOE* and IS have produced conflicting results [16–18], which may be caused by the differences of the methodology used and the populations included.

A stroke belt was found in Northwest China with the high stroke incidence [19]. Many researchers focused on the study of risk genes for IS, but the results are still not sufficient in this area. Therefore, we performed a case–control study in a Northwest China Han population to investigate the association between IS and *APOE* gene polymorphisms.

## Materials and methods

### Subject recruitment

This case–control study recruited 1030 subjects from January, 2011 to December, 2013 in the second hospital of Lanzhou University. The subjects of cases and controls group were enrolled from the department of neurology and physical examination center respectively, both of the two groups included 515 subjects. The 515 subjects in cases group were diagnosed as IS by two senior neurologists according to the criteria of the Chinese Medical Association in 1995 and the criteria amended in the fourth National Cerebrovascular Disease conference, with confirmation on clinical symptoms or signs, laboratory results, and computerized tomography scan (CTS) or magnetic resonance imaging (MRI). The subjects who underwent physical examination from January, 2011 to December, 2013 in The Second Hospital of Lanzhou University and did not have cerebrovascular diseases and other serious neurological diseases were included in the control group. The subjects in control group without IS were performed medical history material collection, physical examination, and head imaging examination (CTs or MRI) to determine the cerebrovascular diseases and other severe neurological diseases. In addition, the patients with severe liver and kidney diseases were also excluded from the participants in the present study. In genotyping process of *APOE*, three DNA samples were not detected successfully, so we excluded them from the following analysis, including two IS patients and one control participant. The average age of cases group (294 males and 219 females) and control group (288 males and 226 females) were 62.26 ± 12.16 and 61.66 ± 13.49 respectively.

Participants completed a series of clinic examinations which included a medical history interview, physical examination, and auxiliary tests. Some risk factors for IS were recorded, including hypertension (a systolic blood pressure ≥140 mmHg or a diastolic blood pressure ≥90 mmHg, and/or patients were receiving antihypertensive treatment), diabetes (fasting serum glucose (GLU) ≥7.0 mmol/l or the use of either insulin or oral hypoglycemic medications), dyslipidemia (fasting serum total cholesterol (TC) ≥5.80 mmol/l, triacylglycerides (TG) ≥1.80 mmol/l, high-density lipoprotein (HDL) ≤0.70 mmol/l, low-density lipoprotein (LDL) ≥3.30 mmol/l), and cardiopath (arrhythmia and coronary artery disease). IS sorting was performed according to the Trial of ORG 10172 in Acute Stroke Treatment (TOAST) classification system [20]. All subjects were Han Chinese, and came from Gansu province in the Northwest of China. There was no kinship among the controls or stroke patients. Informed consent was obtained from all subjects before study. The protocol of the present study was approved by the Ethics Committee of The Second Hospital of Lanzhou University (lzdxyxy20140310).

### Sample size calculation

The prevalence for the ε4 allele in cases and controls was 0.125 and 0.071 respectively [21]. Assuming 90% power and two-sided 5% α, we obtained the minimum sample size 404 in each group. In our study, 515 cases and 515 controls were included, which could meet the minimum sample size requirement.

### Blood sample and DNA extraction

After an overnight fast, venous blood was collected from each subject in cases and controls groups and placed into the vacuum tube coated with EDTA2K. By using TIANamp Blood DNA Kit (DP318) (Tiangen Biotech, Beijing, China), DNA was extracted from blood samples of subjects. The concentration and OD ratio was tested by NanoDrop 2000 (Thermo Fisher Scientific, Wilmington, DE, U.S.A.) for quality inspection of DNA.

### Genotyping

According to the alleles of two single nucleotide polymorphisms of *APOE*, rs429358, and rs7412, the *APOE* genotyping was performed by the MassARRAY iPLEX system (Sequenom, Inc., San Diego, CA, U.S.A.) *After an overnight fast, venous blood was collected from each subject in cases and controls groups and placed into the vacuum tube coated with EDTA2K. By using TIANamp Blood DNA Kit (DP318) (TIANGEN Biotech, Beijing, China), DNA was extracted from blood samples of subjects. The concentration and OD ratio were tested by NanoDrop 2000 (Thermo Fisher Scientific, Wilmington, DE, U.S.A.) for quality inspection of DNA.*(Table 1). In order to control quality, two repetitions and two blank samples were set in each 96-well plate as polymerase chain reaction-negative controls. In genotyping process of *APOE*, three DNA samples were not detected successfully. Missed detection rate for all 1030 DNA samples was 0.29%. So, we excluded them from the following analysis, including two IS patients and one control participant.

**Table 1:** Genotyping of *APOE*

*APOE*	rs429358	rs7412
ε2/ε2	TT	TT
ε2/ε3	TT	TC
ε2/ε4	TC	TC
ε3/ε3	TT	CC
ε3/ε4	TC	CC
ε4/ε4	CC	CC

### Statistical analysis

Data analysis was performed using the SPSS software version 19.0 (IBM, Armonk, New York) and the normality test was conducted using Shapiro–Wilk (SW) test before doing the parametric analysis. The Hardy–Weinberg equilibrium (HWE) was assessed by chi-square test. General information and risk factors between cases and controls group were compared with Student’s *t*-test or Pearson’s *χ*^2^ test, so as to determine the association between *APOE* ε4 allele and risk factors of IS. Univariate and multivariate logistic regression was performed to evaluate distribution differences of *APOE* genotypes and alleles in cases (all IS and subtypes) and controls group after adjusting age, gender, and body mass index (BMI), at the same time the odds ratios (OR) and 95% confidence intervals were calculated to assess the strength of association. All *P* values were two-tailed, and a value of *P*<0.05 was considered statistically significant.

## Results

The two single nucleotide polymorphisms of *APOE*, rs429358 and rs7412, were in HWE in both cases and controls groups (*P*>0.05). The clinical characteristics of cases and controls groups were showed in Table 2. There were no significant differences on average age, male/female ratio, and average BMI between the cases and controls groups. Blood laboratory tests results showed that IS susceptibility was associated with GLU, TC, TG, HDL, and LDL. Comparing the medical history in two groups of subjects, the proportions of hypertension, diabetes, dyslipidemia, and cardiopath were higher in IS groups (*P*<0.01). So, the risk factors for IS indicated in the present study are the levels of GLU, TC, TG, HDL, LDL in blood and medical history of hypertension, diabetes, dyslipidemia, and cardiopath. According to the TOAST classification, the proportions for the five subtypes were 23.20%, 5.26%, 47.17%, 1.75%, and 22.61% respectively, refer to large artery atherosclerosis (LAA), cardio-embolic (CE), small vessel disease (SVD), other determined causes, and undetermined IS respectively.

**Table 2:** Clinical characteristics of patients and controls

Characteristics	IS Cases	Controls	*P* value
Number	513	514	–
Age	62.26 ± 12.16	61.66 ± 13.49	0.452*
Gender (M/F)	294/219	288/226	0.679^†^
BMI (kg/m^2^)	24.83 ± 2.73	24.76 ± 2.83	0.677*
Glu (mmol/l)	5.54 ± 3.46	4.55 ± 0.92	<0.001*
TC (mmol/l)	4.32 ± 1.05	3.65 ± 0.96	<0.001*
TG (mmol/l)	1.50 ± 0.92	1.06 ± 0.59	<0.001*
HDL (mmol/l)	1.25 ± 0.55	1.60 ± 0.38	<0.001*
LDL (mmol/l)	2.59 ± 0.87	1.99 ± 0.61	<0.001*
Hypertension (%)	211(41.13)	115(22.37)	<0.001^†^
Diabetes (%)	139(27.10)	49(9.53)	<0.001^†^
Dyslipidemia (%)	242(47.17)	155(30.16)	<0.001^†^
Cardiopathy (%)	46(8.97)	10(1.95)	<0.001^†^
TOAST			
Large atery atherosclerosis (%)	119(23.20)	–	–
Cadio-embolic (%)	27(5.26)	–	–
Small vessel disease (%)	242(47.17)	–	–
Other determined causes (%)	9(1.75)	–	–
Undetermined (%)	116(22.61)	–	–

*Student’s *t*-test; ^†^Pearson’s *χ*^2^ test. Abbreviations: BMI, body mass index; F, female; Glu, glucose; HDL, high-density lipoprotein; LDL, low-density lipoprotein; M, male; TC, total cholesterol; TG, triglyceride; TOAST, Trial of ORG 10172 in Acute Stroke Treatment.

In Northwest China, *APOE* ε3/ε3 genotype and ε3 allele were predominant in both IS patients and controls, as shown in Table 3. Therefore, ε3/ε3 genotype and ε3 allele were account as references in the following analysis. The results of the comparison for genotypes and alleles distribution differences between cases and controls showed that ε4/ε4 genotype and ε4 allele were associated with IS in this population (ε4/ε4 vs. ε3/ε3, *P*=0.045; ε4 vs. ε3, *P*=0.012). In consideration of the small number of subjects with ε4/ε4 genotype, those with ε2/ε4, ε3/ε4, and ε4/ε4 genotype were merged into ε4-containing genotype group. Compared with controls, the prevalence of ε4-containing genotypes was significantly higher in cases (*P*=0.027), as is consistent with above results.

**Table 3:** Distribution of *APOE* alleles and genotypes

Alleles/Genotypes	Controls (*N*=514)	All IS (*N*=513)	*P* value	OR (95%CI)
Alleles				
ε2	88(8.56)	76(7.41)	0.461	0.886(0.642–1.222)
ε3	866(84.24)	842(82.07)	–	–
ε4	74(7.20)	108(10.53)	**0.012**	1.491(1.093–2.035)
Genotypes				
ε2/ε2	5(0.97)	3(0.58)	0.560	0.651(0.154–2.756)
ε2/ε3	70(13.62)	63(12.28)	0.765	0.945(0.652–1.370)
ε2/ε4	8(1.56)	7(1.36)	0.891	0.931(0.333–2.600)
ε3/ε3	366(71.21)	347(67.64)	–	–
ε3/ε4	64(12.45)	85(16.57)	0.067	1.396(0.977–1.995)
ε4/ε4	1(0.19)	8(1.56)	**0.045**	8.449(1.050–67.999)
ε4 containing	73(14.20)	100(19.49)	**0.027**	1.453(1.044–2.023)

During the further analysis, the results indicated the association between *APOE* gene polymorphisms and five subtypes of IS (Table 4). In LAA subtype, a significant difference was found between cases and controls in the distribution of *APOE* ε4/ε4 genotypes and ε4 allele. In addition, ε2 allele played a protective role against such type of IS, which was not found in total IS group. In SVD subtype, there was only showed a higher proportion of ε4/ε4 genotype in cases group than controls group but not with ε4 allele. With absence of ε4/ε4 genotype, undermined subtype was correlated with ε4 allele, ε3/ε4 genotype, and ε4-containing genotypes. In other two classes, no association was found between *APOE* gene polymorphisms and disease susceptibility.

**Table 4:** Distribution of *Apo E* alleles and genotypes in IS subtypes

Alleles/Genotypes	Controls *N* (%)	LAA		CE		SVD		OTHER		Undetermined	
		*N* (%)	*P* value OR (95%CI)	*N* (%)	*P* value OR (95%CI)	*N* (%)	*P* value OR (95%CI)	*N* (%)	*P* value OR (95%CI)	*N* (%)	*P* value OR (95%CI)
Alleles											
ε2	88	10	**0.044**	3	0.445	40	0.945	2	0.588	21	0.651
	(9.92)	(4.20)	**0.500 (0.254**–**0.983)**	(5.56)	0.629 (0.192–2.065)	(8.26)	0.986 (0.666–1.462)	(11.11)	1.516 (0.336–6.832)	(9.05)	1.123 (0.679–1.857)
ε3	866	201	–	47	–	397	–	13	–	184	–
	(82.78)	(84.45)	1.000	(87.04)	1.000	(82.02)	1.000	(72.22)	1.000	(79.31)	1.000
ε4	74	27	**0.047**	4	0.973	47	0.109	3	0.135	27	**0.028**
	(7.30)	(11.34)	**1.614 (1.007**–**2.587)**	(7.14)	0.982 (0.344–2.807)	(9.71)	1.372 (0.932–2.019)	(16.67)	2.665 (0.738–9.624)	(11.64)	**1.694 (1.059**–**2.712)**
Genotypes											
ε2/ε2	5	0	–	1	0.232	2	0.841	0	–	0	–
	(0.97)	(0.00)	–	(3.70)	3.894 (0.420–36.147)	(0.83)	0.844 (0.161–4.425)	(0.00)	–	(0.00)	–
ε2/ε3	70	10	0.176	1	0.172	33	0.848	2	0.258	17	0.444
	(13.62)	(8.40)	0.613 (0.302–1.245)	(3.70)	0.244 (0.032–1.848)	(13.64)	1.045 (0.664–1.647)	(22.22)	2.702 (0.482–15.143)	(14.66)	1.259 (0.698–2.270)
ε2/ε4	8	0	–	0	–	3	0.796	0	–	4	0.166
	(1.56)	(0.00)	–	(0.00)	–	(1.24)	0.838 (0.219–3.204)	(0.00)	–	(3.45)	2.392 (0.697–8.210)
ε3/ε3	366	85	–	21	–	165	–	4	–	72	–
	(71.21)	(71.43)	1.000	(77.78)	1.000	(68.18)	1.000	(44.44)	1.000	(62.07)	1.000
ε3/ε4	64	21	0.209	4	0.914	34	0.521	3	0.070	23	**0.033**
	(12.45)	(17.65)	1.425 (0.820–2.478)	(14.81)	1.063 (0.352–3.211)	(14.05)	1.161 (0.735–1.835)	(33.33)	4.126 (0.892–19.095)	(19.83)	**1.806 (1.049-3.111)**
ε4/ε4	1	3	**0.017**	0	–	5	**0.028**	0	–	0	-
	(0.19)	(2.52)	**16.525 (1.657–164.773)**	(0.00)	–	(2.07)	**11.298 (1.306–97.72)**	(0.00)	–	(0.00)	-
ε4 containing	73	24	0.169	4	0.910	42	0.277	3	0.095	27	**0.017**
	(14.20)	(20.17)	1.445 (0.855–2.441)	(14.81)	0.939 (0.312–2.823)	(17.36)	1.265 (0.828–1.932)	(33.33)	3.678 (0.797–16.987)	(23.28)	1.868 (1.120-3.115)

Abbreviations: CE, cardio-embolic; LAA, large artery atherosclerosis; SVD, small vessel disease.

In order to further illuminate the underlying mechanisms for *APOE* and IS association, analysis was performed to explore the association between ε4-containing genotypes and clinical characteristics in subjects (Table 5). TC and LDL levels in blood were higher in IS patients with ε4 allele compared with controls. In controls group, besides the TC and LDL levels of blood, it was also showed that TG level in blood was higher in subjects with ε4 allele. After combining cases and controls together, the results showed that the TC and LDL levels in blood were higher in people with ε4 allele. Furthermore, the proportion of subjects with cardiopath history was higher in groups with ε4 allele compared with subjects without ε4 allele. Some clinical information did not relate with *APOE* gene polymorphisms as shown in the present study, including age, gender, BMI, HDL, and history of hypertension, diabetes, dyslipidemia.

**Table 5:** Association of ε4-containing genotypes with clinical characteristics in IS patients

Characteristics	Cases		*P* value	Controls		*P* value	All		*P* value
	With ε4	Without ε4		With ε4	Without ε4		With ε4	Without ε4	
Number	100	413	–	73	441	–	173	854	–
Age	64.20 ± 12.19	61.79 ± 12.13	0.452	62.23 ± 12.97	61.56 ± 13.59	0.693	63.37 ± 12.53	61.67 ± 12.89	0.113
Gender (M/F)	58/42	236/177	0.876	39/34	249/192	0.628	97/76	485/369	0.861
BMI (kg/m^2^)	24.90 ± 2.74	24.82 ± 2.73	0.789	24.91 ± 2.92	24.73 ± 2.80	0.618	24.90 ± 2.81	24.77 ± 2.77	0.574
Glu (mmol/l)	5.16 ± 1.70	5.63 ± 3.76	0.226	4.52 ± 0.84	4.56 ± 0.94	0.741	4.89 ± 1.43	5.08 ± 2.75	0.389
TC (mmol/l)	4.59 ± 1.05	4.25 ± 1.04	**0.003**	3.89 ± 1.04	3.60 ± 0.98	**0.032**	4.30 ± 1.10	3.92 ± 1.06	**4.47E−5**
TG (mmol/l)	1.50 ± 0.75	1.50 ± 0.96	0.996	1.21 ± 0.76	1.02 ± 0.48	**0.048**	1.38 ± 0.77	1.26 ± 0.79	0.061
HDL (mmol/l)	1.24 ± 0.45	1.25 ± 0.58	0.779	1.56 ± 0.40	1.60 ± 0.37	0.355	1.37 ± 0.46	1.43 ± 0.51	0.143
LDL (mmol/l)	2.81 ± 0.83	2.54 ± 0.88	**0.005**	2.16 ± 0.85	1.94 ± 0.61	**0.036**	2.54 ± 0.90	2.23 ± 0.81	**4.51E−5**
Hypertension (%)	44 (44.00)	167 (40.44)	0.516	18 (24.66)	97 (22.00)	0.163	62 (35.83)	264 (30.91)	0.204
Diabetes (%)	21 (21.00)	118 (28.57)	0.126	9 (12.33)	40 (9.07)	0.380	30 (17.34)	158 (18.50)	0.719
Dyslipidemia (%)	52 (52.00)	190 (46.00)	0.281	17 (23.29)	138 (31.29)	0.167	69 (39.88)	328 (38.41)	0.716
Cardiopathy (%)	14 (14.00)	32 (7.75)	0.050	2 (2.74)	8 (1.81)	0.596	16 (9.25)	40 (4.68)	**0.016**

Abbreviations: BMI, body mass index; F, female; Glu, glucose; HDL, high-density lipoprotein; LDL, low-density lipoprotein; M, male; TC, total cholesterol; TG, triglyceride; TOAST, Trial of ORG 10172 in Acute Stroke Treatment.

In order to determine whether the clinical variables and ε4-containing genotypes were independent risk factors for IS, a multivariate logistic regression analysis was performed using three models. The results were shown in Table 6. ε3/ε3 genotype and ε3 allele were account as references in the following analysis. The three models included different independent variables. The six genotypes were included in Model 1, Glu, TC, TG, HDL, LDL, hypertension, and cardiopathy were statistically significant (all *P*<0.05) while the six genotypes were all non-significant (all *P*>0.05). In Model 2, we combined all the genotypes with ε4, including ε2/ε4, ε3/ε4, and ε4/ε4, the similar results to Model 1 were obtained. *APOE* allele was included in Model 3, including ε2, ε3, and ε4. Diabetes and dyslipidemia were also statistically significant like the other biochemical parameters mentioned in the previous two models (all *P*<0.05), and the three alleles showed no statistical difference (all *P*>0.05). The results suggested that the *APOE* gene was an influence factor for IS, but was not an independent influence factor (Table 6).

**Table 6:** Multivariable logistic regression analysis for risk factors of ischemic stroke

Characteristics	Model 1		Model 2		Model 3	
	*P* value	OR (95%CI)	*P* value	OR (95%CI)	*P* value	OR (95%CI)
Age	0.070	1.011 (0.999–1.023)	0.064	1.011 (0.999–1.023)	**0.009**	1.011 (1.003–1.020)
Gender	0.990	0.998 (0.733–1.359)	1.000	0.998 (0.735–1.362)	0.982	0.998 (0.802–1.241)
BMI	0.768	0.992 (0.940–1.047)	0.817	0.994 (0.942–1.049)	0.896	0.997 (0.960–1.036)
Glu	**<0.001**	1.530 (1.288–1.817)	**<0.001**	1.525 (1.285–1.811)	**<0.001**	1.527 (1.353–1.724)
TC	**0.012**	1.334 (1.066–1.669)	**0.011**	1.339 (1.071–1.675)	**<0.001**	1.344 (1.149–1.573)
TG	**0.022**	1.352 (1.045–1.750)	**0.024**	1.343 (1.040–1.736)	**0.001**	1.344 (1.122–1.611)
HDL	**<0.001**	0.198 (0.133–0.295)	**<0.001**	0.197 (0.132–0.293)	**<0.001**	0.198 (0.149–0.262)
LDL	**<0.001**	1.990 (1.496–2.648)	**<0.001**	1.995 (1.500–2.654)	**<0.001**	1.969 (1.613–2.404)
Hypertension	**0.009**	1.574 (1.123–2.208)	**0.009**	1.569 (1.120–2.199)	**<0.001**	1.602 (1.264–2.030)
Diabetes	0.053	1.609 (0.993–2.607)	0.051	1.615 (0.997–2.615)	**0.007**	1.602 (1.141–2.250)
Dyslipidemia	0.129	0.760 (0.533–1.083)	0.128	0.760 (0.533–1.082)	**0.028**	0.756 (0.589–0.971)
Cardiopathy	**0.023**	2.489 (1.131–5.476)	**0.022**	2.515 (1.144–5.526)	**0.001**	2.488 (1.429–4.332)
*APOE* genotype						
ε3/ε3	1.000		1.000			
ε2/ε2	0.971	0.965 (0.139–6.697)	0.976	0.971 (0.140–6.760)		
ε2/ε3	0.400	1.215 (0.772–1.910)	0.396	1.217 (0.774–1.913)		
ε2/ε4	0.429	0.626 (0.197–1.995)				
ε3/ε4	0.739	1.078 (0.693–1.677)				
ε4/ε4	0.518	2.096 (0.222–19.783)				
ε4-containing			0.856	1.039 (0.685–1.576)		
*APOE* allele						
ε3					1.000	
ε2					0.678	1.086 (0.736–1.602)
ε4					0.844	1.039 (0.709–1.523)

Abbreviations: BMI, body mass index; F, female; Glu, glucose; HDL, high-density lipoprotein; LDL, low-density lipoprotein; M, male; TC, total cholesterol; TG, triglyceride; TOAST, Trial of ORG 10172 in Acute Stroke Treatment.

**Model 1** includes six different *APOE* genotype; **Model 2** includes ε4-containing gene; **Model 3** includes three different *APOE* alleles.

## Discussion

To date, studies of the association between IS and *APOE* gene polymorphisms have been performed in some cohorts and yielded somewhat inconsistent results. In the present study, we found that *APOE* gene polymorphisms were associated with IS susceptibility in a Northwest China Han people. It is consistent with a large meta-analysis, which showed that such relation was more distinct in Asia population [10]. However, in a large sample study conducted by ARIC (Atherosclerosis Risk in Communities), involves 15792 men and women, aged 45–64 years, the results showed that *APOE* was not a risk factor for incident of IS [15], which is opposite to our conclusion. The differences of age, sample size, and ethnicities in studies may also account for the disagreement. The mean age of our study is 10 years older than that in ARIC study.

In LAA and SVD subtypes, genetic factors seem to be more important than other IS subtypes [22,23]. It was also confirmed in our study on the *APOE* and IS association. A research showed a clear association of *APOE* with carotid intima-media thickness [24]. It is possible that *APOE* influence LAA, for which carotid intima-media thickness is an informative intermediate phenotype. Apart from the relationship between *APOE* ε4 allele and IS, in LAA, *APOE* ε2 allele played a protector role against IS. A study found such weak protective effects in black women [16]. Besides, the apparent relation between *APOE* and undetermined subtype was found in the present study. Considering the lack of precise examination for cerebrovascular disease and two or more subtypes mix, the classification was not accurate enough. From this perspective, the association between *APOE* and undetermined subtype might be a false appearance for such association with other subtypes. On the other hand, the further studies still need to perform to explore the mechanisms underlying this association.

Traditional risk factors for IS were affected by *APOE* gene polymorphism indicated in the present study, including TC, TG, and LDL in blood. It was found that TC, TG, and LDL levels of serum were higher in the patients with ε4 allele, which coincides with previous studies [25–27]. The nexus of blood lipid level and *APOE* genotypes was found in all subjects. And compared with controls, the levels of blood TC, TG, and LDL were higher in cases group. It can be derived that *APOE* gene polymorphism takes effect on IS incidence through the influence on plasma lipid. In the present study, the correlation of cardiopath and *APOE* variants was found in all subjects. The cardiopath history mentioned in the present study included coronary heart disease and arrhythmia. It is confirmed in some meta-analysis that carriers of ε4 allele have increased risk for coronary heart disease in Chinese [28,29]. And it was showed that the *APOE* variants result in a 2-fold or greater increased risk for coronary artery disease, myocardial infarction, and ventricular fibrillation [30]. Researches showed that APOE ε4 allele was associated with BMI, hypertension, and diabetes [31–33]. But the present study did not show such nexuses. A study in a cognitively normal aging Han Chinese population showed that there was no correlation between *APOE* genotypes and serum levels of GLU [25], which is consistent with the present study. All in all, the results of analysis for association between *APOE* ε4 allele and some traditional risk factors of IS showed that plasma lipid level was affected by *APOE* variants. Given that high levels of blood TC, TG, and LDL were related to IS incidence, the relations of *APOE* ε4 allele to IS might be attributable, at least in part, to the effect on lipid level. However, other mechanisms underlying *APOE* and IS association are still undetermined.

The present study has several strengths and weaknesses. One hand, with a relatively large sample subjects who were homogeneous ethnicity and geographic region, complete and accurate information collection, and a high throughput platform for *APOE* genotyping, our study is creditable and valid. On the other hand, selection bias cannot be protected against thoroughly in such a case–control study. Also, in the present study, the age and gender were not exactly matched in the two groups, which may reduce the effectiveness of study and introduce selection bias, but the age and gender were equally comparable in the two groups (*P*>0.05). Therefore, further researches are needed to verify the association between *APOE* and IS in Northwest China. Moreover, the underlying mechanisms are also need to study in depth.

In summary, it appears that *APOE* gene is a risk factor for IS in a Northwest China Han population included in the present study, especially for some subtypes, LAA, SVD, and undetermined subgroups. Blood lipid level is higher in subjects with ε4 allele. For some limits in our study, replication of study on *APOE* and IS association will conducive to further elucidate the role of *APOE* in IS incidence.

## Abbreviations

APOE: Apolipoprotein E
BMI: body mass index
CE: cardio-embolic
GLU: glucose
HDAC9: histone deacetylase 9
HWE: Hardy–Weinberg equilibrium
IS: Ischemic stroke
LAA: large artery atherosclerosis
LDL: low-density lipoprotein
MRI: magnetic resonance imaging
MTHFR: methylenetetrahydrofolate reductase
SVD: small vessel disease
TC: total cholesterol
TG: triacylglycerides
TOAST: Trial of ORG 10172 in Acute Stroke Treatment
